The article "Human hematopoietic signal peptide-containing secreted 1 (hHSS1) modulates genes and pathways in glioma: implications for the regulation of tumorigenicity and angiogenesis" was published in 2014. Journal: BMC Cancer.

# Human hematopoietic signal peptide-containing secreted 1 (*h*HSS1) modulates genes and pathways in glioma: implications for the regulation of tumorigenicity and angiogenesis

**DOI:** 10.1186/1471-2407-14-920

**Published:** 2014-12-06

**Authors:** Katiana S Junes-Gill, Chris E Lawrence, Christopher J Wheeler, Ryan Cordner, Tristan G Gill, Vernon Mar, Liron Shiri, Lena A Basile

**Affiliations:** Neumedicines Inc., 133 N Altadena Dr. #310, Pasadena, CA 91107 USA; Department of Neurosurgery, Maxine Dunitz Neurosurgical Institute, Cedars-Sinai Medical Center, 8700 Beverly Blvd., Davis Rm. 2097, Los Angeles, CA 90048 USA; Ingenuity Systems, 1700 Seaport Blvd, 3rd Floor, Redwood City, CA 94063 USA

**Keywords:** Glioma, Microarray, *h*HSS1, C19orf63, Cell migration, Cell invasion, Angiogenesis, TCGA database, U87, A172

## Abstract

**Background:**

Human Hematopoietic Signal peptide-containing Secreted 1 (*h*HSS1) is a truly novel protein, defining a new class of secreted factors. We have previously reported that ectopic overexpression of *h*HSS1 has a negative modulatory effect on cell proliferation and tumorigenesis in glioblastoma model systems. Here we have used microarray analysis, screened glioblastoma samples in The Cancer Genome Atlas (TCGA), and studied the effects of *h*HSS1 on glioma-derived cells and endothelial cells to elucidate the molecular mechanisms underlying the anti-tumorigenic effects of *h*HSS1.

**Methods:**

Gene expression profiling of human glioma U87 and A172 cells overexpressing *h*HSS1 was performed. Ingenuity® iReport™ and Ingenuity Pathway Analysis (IPA) were used to analyze the gene expression in the glioma cells. DNA content and cell cycle analysis were performed by FACS, while cell migration, cell invasion, and effects of *h*HSS1 on HUVEC tube formation were determined by transwell and matrigel assays. Correlation was made between *h*HSS1 expression and specific genes in glioblastoma samples in the TCGA database.

**Results:**

We have clarified the signaling and metabolic pathways (i.e. role of BRCA1 in DNA damage response), networks (i.e. cell cycle) and biological processes (i.e. cell division process of chromosomes) that result from *h*HSS1effects upon glioblastoma growth. U87-overexpressing *h*HSS1 significantly decreased the number of cells in the G0/G1 cell cycle phase, and significantly increased cells in the S and G2/M phases (*P* < 0.05). U87-overexpressing *h*HSS1 significantly lost their ability to migrate (*P* < 0.001) and to invade (*P* < 0.01) through matrigel matrix. *h*HSS1-overexpression significantly decreased migration of A172 cells (*P* < 0.001), inhibited A172 tumor-induced migration and invasion of HUVECs (*P* < 0.001), and significantly inhibited U87 tumor-induced invasion of HUVECs (*P* < 0.001). Purified *h*HSS1 protein inhibited HUVEC tube formation. TCGA database revealed significant correlation between *h*HSS1 and *BRCA2* (r = −0.224, *P* < 0.0005), *ADAMTS1* (r = −0.132, *P* <0.01) and endostatin (r = 0.141, *P* < 0.005).

**Conclusions:**

*h*HSS1-overexpression modulates signaling pathways involved in tumorigenesis. *h*HSS1 inhibits glioma-induced cell cycle progression, cell migration, invasion and angiogenesis. Our data suggest that *h*HSS1 is a potential therapeutic for malignant glioblastoma possessing significant antitumor and anti-angiogenic activity.

## Background

Human Hematopoietic Signal peptide-containing Secreted 1 (*h*HSS1) is a truly novel protein, as it has no homology to any known protein, or protein domain. Consequently, *h*HSS1 defines a new class of secreted factors. Although little is known about *h*HSS1, there is evidence that *h*HSS1 is one of the glucose-responsive genes with both mRNA and protein secretion being regulated by glucose [1]. As such, it is speculated that *h*HSS1 could be associated with the functions of pancreatic islets, specifically beta-cells [1]. Recently, *h*HSS1 was identified as endoplasmic reticulum (ER) membrane protein complex subunit 10 (EMC10), one of the components of ER associated degradation (ERAD), an ubiquitin and proteasome dependent process [2]. The mouse orthologue of *h*HSS1 (C19orf63) is the only gene that is highly expressed in mice with the 22q11.2 microdeletion, an animal model used to study the association between 22q11.2 microdeletion and a strong risk for schizophrenia development [3]. Up-regulation of Mirta 22, the mouse orthologue of *h*HSS1, was shown to be responsible for abnormal neuronal morphology through the inhibition of neuronal connectivity, again linked to schizophrenia susceptibility and cognitive deficit [3]. It was also verified that Mirta 22 expression was purely neuronal and located in the Golgi apparatus [3]. We have previously demonstrated that ectopic overexpression of *h*HSS1 has a negative modulatory effect on cell proliferation and tumorigenesis, in both *in vitro* and *in vivo* murine model of glioblastoma [4]. However, the molecular mechanism by which *h*HSS1 suppresses cell proliferation and tumorigenesis has yet to be defined.

The National Cancer Institute (NCI) estimates that 22,340 new cases and 13,110 deaths from brain and other nervous system cancers occurred in US in 2011. Malignant gliomas are the most common and most aggressive primary brain tumor, accounting for more than half of the new cases of primary malignant brain tumors diagnosed each year in US [5]. Given the fatal effect of most neurological and brain cancers, novel approaches are needed to increase survival rate of patients diagnosed with these diseases. Contemporary treatment modalities do not substantially increase the survival rate and generally are not curative. There is a critical need to elucidate novel pathways and factors involved in the inhibition of tumor growth in glioma, in order to facilitate the development of novel anti-tumoral therapeutics that may be key in controlling and, eradicating malignant glioma. Identifying and characterizing novel proteins, such as *h*HSS1, opens up the possibility of discovering such novel biological functions and pathways. Thus, it is critical to characterize and dissect the anti-tumoral effect of *h*HSS1.

Here we have defined the global expression profile of A172 and U87 human glioma-derived cells overexpressing *h*HSS1 to gain insights into the mechanism by which *h*HSS1 acts on glioma cells and to further elucidate its function. For this purpose, we used microarray analysis to determine cellular transcriptional changes in response to 96–120 hours of *h*HSS1 overexpression in stably transfected cells [4]. Focused analysis of these time points would allow the identification of early *h*HSS1 regulated genes involved in the cytostatic effect exerted by *h*HSS1 in A172 and U87 human glioma-derived cells. cDNA microarray analysis might be useful for the elucidation of the key factors in tumorigenesis, and facilitate identification of genes involved in pathways related to *h*HSS1. This could lead to significant progress in the treatment of human disease by defining new therapeutics and novel molecular targets, particularly in glioma. Analysis of the TCGA database and the effect of *h*HSS1 on cell cycle, migration and invasion of glioma-derived cells, as well as the effect of *h*HSS1 on the angiogenic properties of HUVEC are described.

## Methods

### Cell culture

A172 glioma cell lines (ATCC, Manassas, VA, USA) were cultured in DMEM supplemented with 10% FBS (Life technologies, Grand Island, NY, USA). The human U87 glioma cell line (ATCC HTB-14) was maintained in alpha-MEM (ATCC, Manassas, VA, USA) supplemented with 10% FBS. HUVECs (LONZA, Allendale, NJ, USA) were maintained in EGM (LONZA, Allendale, NJ, USA).

### Stable transfection

The glioblastoma-derived A172 and U87 cell lines were stably transfected with *h*HSS1 as previously described [4]. Stable clones were maintained with 500ug ml^−1^ of G-418 (Invitrogen, Carlsbad, CA, USA) added to the cultures. The pcDNA3.1 construct used to stably express *h*HSS1 had a 6-His tag in-frame fused at the C-terminal of the *h*HSS1 gene.

### Transcript expression profiling using microarray

GeneChip Human Gene 1.0 ST Array (*Affymetrix*, Santa Clara, CA, USA) was used to obtain transcript expression profiles in wild type (non-transfected), mock stable-transfected (pcDNA3.1 empty vector) and *h*HSS1-stable-transfected (pcDNA3.1-*h*HSS1) U87 and A172 cells. U87 cells (4 × 10^5^) were cultured in duplicate in 10 cm plates and incubated at 37°C, 5% CO_2_. After 5 days, cells were harvested by trypsinization and viability determined by trypan blue exclusion. A172 cells (2 × 10^5^) were plated in triplicate in 10 cm plates and after 4 days the cells were harvested and counted. The expression profile of one clone of U87 cells and two clones of A172 cells (C#7 and C#8) expressing *h*HSS1 was evaluated. Expression of *h*HSS1 mRNA on stable clones was confirmed using qRT-PCR prior to microarray analysis. Total RNA was isolated using the RNeasy minikit (Qiagen, Valencia, CA, USA). During the RNA purification process samples were treated with DNAse on the column before washing with buffer RPE. RNA characterization and chip analysis was carried out at the Functional Genomics Core of the City of Hope (Duarte, CA, USA) and at the Core Facility of Children’s Hospital Los Angeles (Los Angeles, CA, USA). Technical replicates of U87 RNA samples were evaluated in triplicates and A172 cells were evaluated in biological triplicates. Expression values were determined using dChip (July 9, 2009 build) or Partek software (St. Louis, MO, USA). The data discussed in this publication have been deposited in NCBI's Gene Expression Omnibus [6] and are accessible through GEO Series accession number GSE61780 (http://www.ncbi.nlm.nih.gov/geo/query/acc.cgi?acc=GSE61780).

### Network and pathways analysis

Ingenuity Pathway Analysis (IPA, Ingenuity® Systems, http://www.ingenuity.com, Redwood City, CA, USA) was done using differentially expressed genes (DEGs) with *P* < 0.001 with at least a 1.3 (A172 cells) and 1.5 (U87 cells) fold-change between *h*HSS1 expressing cells and control. For Ingenuity® iReport analysis (Ingenuity® Systems, http://www.ingenuity.com, Redwood City, CA, USA), gene expression was considered significant at *P* < 0.05 and a fold change cutoff of 2 (U87 cells) and 1.5 (A172 cells) were deemed significant. A lower cutoff was chosen for A172 cells because of the small number of DEGs. The scores generated by the network and pathway analysis are derived from a *P*-value and indicates the likelihood of the focus gene connectivity to be due to random chance. A score of 2 indicates that there is a 1 in 100 chance that the focus genes are together in a network due to random chance. Therefore, scores of 2 or higher have at least a 99% confidence of not being generated by random chance alone.

### qRT-PCR

Validation of DEGs from the microarray analysis was done by quantitative RT-PCR. cDNA synthesis was performed by reverse transcription of total RNA using Transcriptor First Strand cDNA Synthesis Kit (Roche, Indianapolis, IN, USA). qRT-PCR was performed using gene-specific primers and hydrolysis probes (Biosearch Technologies, Petaluma, CA, USA) and LightCycler 480 Probes Master Kit reagents (Roche, Indianapolis, IN, USA). All reactions were performed in triplicate, using a total of 18 μl/well with primer concentration of 100 nM, in a LightCycler 480 System (Roche, Indianapolis, IN, USA). Five different target genes were selected for each cell line. Each target was normalized to RPL32 housekeeping gene. Relative expression was calculated using LightCycler 480 Software 1.5 version (Roche, Indianapolis, IN, USA). Fold-change was determined by the ratio between cells overexpressing *h*HSS1/cells overexpressing empty vector, and represented by fold-change if >1 and −1/fold-change if <1. Data were represented as mean values of biological triplicates (A172) and technical triplicates (U87).

### Cell cycle analysis

Exponentially growing U87 cells at growth curve day 4 and A172 cells at growth curve day 5 [4] were harvested by trypsinization and stained with 50 μg/ml propidium iodide, 100 μg/mL RNAase DNase-free (Roche, Indianapolis, IN, USA). DNA content and cell cycle distribution were analyzed by FACS (Beckman Counter, EPICS-XL, Fullerton, CA, USA). Two independent experiments were performed.

### Transwell migration assay

BD BioCoat transwell chambers (BD Biosciences, Bedford, MA, USA) with 8-μM pore size PET membrane inserts for 24-well plates were used according to the manufacturer instructions. Briefly, 5 × 10^4^ cells in serum free medium (DMEM or EMEM) were plated in the upper well of the transwell chambers, whereas medium supplemented with 10% FBS was added to the lower chamber as the chemoattractant. Following a 22 h incubation, the cells on the upper side of the inserts were removed using a cotton swab. The inserts were fixed in cold methanol and stained with hematoxylin and eosin (H&E, Sigma-Aldrich, St. Louis, MO, USA). The number of migrated cells attached to the other side of the insert was counted from 9 random fields using a BX41 Olympus microscope (Center Valley, PA, USA) equipped with 20X objective lens. Pictures were taken at a magnification of 200× using a DP73 camera (Olympus, Center Valley, PA, USA) mounted on the microscope. Two independent experiments were done in duplicates. We performed a co-culture assay to verify a glioblastoma cell-induced migration of HUVEC cells. Briefly, U87 or A172 cells (2.5 × 10^5^) were seeded in the outer chamber of a 24-well plate with DMEM or EMEM supplemented with 2% FBS. Cells were allowed to adhere for 8 h at 37°C, 5% CO_2_. After that, media was changed to serum-free media containing 0.1% BSA and incubated overnight at 37°C, 5% CO_2_ for conditioned media production. Next day, 2.5 × 10^4^ HUVEC cells (1:10 ratio of glioblastoma cells) in serum-free media containing 0.1% BSA were seeded in the upper chamber. After 24 h, migrated cells from 21 fields were counted. Pictures were taken at a magnification of 200×. Two independent experiments were performed in duplicates.

### Transwell invasion assay

Invasion assays were performed using BD BioCoat Matrigel Invasion Chambers (BD Biosciences, San Jose, CA, USA) according to the manufacturer instructions. Briefly, A172 or U87 (5 × 10^4^) cells in serum free medium (DMEM or EMEM) were plated in the upper well of the transwell chambers, whereas medium containing 10% FBS was placed into the lower chamber. The cells were allowed to invade thought the matrix for 24 h. After that, the cells growing on matrigel in the upper chamber were removed using a cotton swab. The inserts were fixed in cold methanol and stained with H&E. The number of invaded cells attached to the other side of the insert was counted from 9 random fields. Pictures were taken at a magnification of 200×. Two independent experiments were done in duplicates. Co-culture assay to verify a glioblastoma cell-induced invasion of HUVEC cells was performed. This experiment was done using the same conditions as mentioned above for the HUVEC co-culture migration assay, with the exception that inserts coated with matrigel were used. Two independent experiments were done in duplicate.

### Angiogenesis assay

The angiogenesis *in vitro* assay was conducted in 96-well plates coated with 50 ul of ECMatrix™ (Millipore, Billerica, MA, USA) following the manufacturer’s instructions. HUVEC cells (2.5 × 10^4^ cells/well) were treated with purified *h*HSS1-his or vehicle control (PBS 1X) in EGM (LONZA, Allendale, NJ, USA) containing 1.2-1.5% FBS. Briefly, cells were pre-treated with 500 nM and 200 nM of *h*HSS1-his or vehicle control for 3 h at 37°C, 5% CO_2_. Vehicle control was diluted following the protein dilution scheme. HUVECs were then plated onto matrigel-coated plates and incubated at 37°C, 5% CO_2_ for 8 h to allow tube formation. After that, cells were stained with 0.5% crystal violet diluted in 50% ethanol and 5% formaldehyde and tube formation was evaluated. Two independent experiments were done in duplicate.

### TCGA database analysis

We selected 428 glioblastoma (GBM) samples from the TCGA database that had both level 3 UNC Agilent G4502A microarray gene expression data and corresponding clinical information. A list of 12 genes was prospectively selected to correlate with *h*HSS1 gene expression. These genes were: *ADAMTS1, APLN, BRCA1, BRCA2, CDKN2A, COL18A1* (endostatin), *EGFR, JAM2, MMP9, RAD51, STAT3*, and *THBS1. h*HSS1 expression was compared with the selected genes using pairwise Pearson correlations, with r values ≥ 0.128 being considered significant. High and low *h*HSS1 expression (Log2-transformed) was subdivided by the median expression level of the GBM cohort, and mean gene expression levels between high and low *h*HSS1 expression cohorts for each of the 12 genes was compared by the two-tailed Student’s t-test. Differences were considered statistically significant when *P* < 0.01.

### Statistical analysis

Differences among groups in the cell cycle analysis were determined by one way ANOVA with Tukey’s test for pairwise post-hoc comparisons. Differences were considered statistically significant when *P* < 0.05. For the migration and invasion assays, two-tailed Student’s t-test was performed to establish the statistical significance of differences between control cells and *h*HSS1-expressing cells. Differences were considered statistically significant when *P* < 0.01.

## Results

### Overview of microarray analysis

Exponentially growing A172 and U87 cells were harvested after 4 and 5 days, respectively. *h*HSS1-expressing cells and control cells were at confluence 40-80% when harvested. Trypan blue analysis of the number of viable cells showed a significant anti-proliferative effect in both cell lines expressing *h*HSS1 as compared to the control cells (A172/U87 wild-type and A172/U87-pcDNA3.1 empty vector). This supports our previously reported data [4].

Total RNA was analyzed on *Affymetrix* GeneChip Human Gene 1.0 ST Array which contains 28,869 genes represented by approximately 26 probes spread across the full length of the gene. These genes, along with their fold-change values, served as input to Ingenuity® iReport or IPA (Ingenuity® Systems, http://www.ingenuity.com). Canonical pathways are shown as depicted by Ingenuity® iReport or IPA. A right-tailed Fisher's exact test was used to identify over-represented functions/canonical pathways. The *P*-values derived through these analyses were based on: 1) total number of functions/canonical pathways eligible molecules that participate in that annotation; 2) total number of knowledge base molecules known to be associated with that function; 3) total number of functions/canonical pathways eligible molecules, and 4) total number of genes in the reference set.

### Up-regulated and down-regulated genes in *h*HSS1-overexpressing A172 and U87 cells

With a cutoff value of a 2 fold change (FC), expression of 1,034 genes was significantly altered when *h*HSS1 was overexpressed in U87 cells (Table 1 and Table 2). The molecules *JUN*, *CDK1*, *VEGFA* and *FOS* showed the highest connectivity ranking. The most down and up-regulated genes were functionally heterogeneous, among them were transcriptional regulators (*ANKRD1*, *MYBL2*), growth factors (*GDF15, PGF*) enzymes (*SLFN11, DHCR24, FBXO32, GCNT3*), transporters (*ATP6V0D2*), phosphatases (*ACPP, PTPRF*), peptidases (*ADAMT55*), cytokines (*IL1RN, IL1A*), kinases (*PDK3, RSPO3*), G-protein coupled receptors (*GPR155, C3AR1*) and transmembrane receptors (*IL13RA2*). There were many transcripts represented that did not have any known protein subcellular localization (*CT45A5, PNLIPRP3, LOC654433, LOC151760, ANO3, MT1M, GLB1L2, FAM115C, C4orf49, FAM111B, FAM70A*) (Table 1 and Table 2).

**Table 1:** **21 most up-regulated genes following** ***h*** **HSS1 overexpression in U87 cells**

Symbol	Gene name	FC
**IL13RA2**	Interleukin 13 Receptor, Alpha 2	112.836
**CT45A5**	Cancer/testis Antigen Family 45, Member A5	37.258
**ATP6V0D2**	Atpase, H+ Transporting, Lysosomal 38 kda, V0 Subunit D2	17.409
**C3AR1**	Complement Component 3a Receptor 1	13.828
**IL1RN**	Interleukin 1 Receptor Antagonist	12.769
**PNLIPRP3**	Pancreatic Lipase-related Protein 3	11.422
**LOC654433**	Hypothetical Loc654433	11.361
**LOC151760**	Hypothetical Loc151760	10.637
**FAM198B**	Family with Sequence Similarity 198, Member B	8.365
**GDF15**	Growth Differentiation Factor 15	8.017
**ANKRD1**	Ankyrin Repeat Domain 1 (Cardiac Muscle)	7.661
**FBXO32**	F-box Protein 32	7.469
**RSPO3**	R-spondin 3 Homolog (Xenopus Laevis)	7.223
**NR0B1**	Nuclear Receptor Subfamily 0, Group B, Member 1	6.862
**IL1A**	Interleukin 1, Alpha	6.842
**GCNT3**	Glucosaminyl (N-acetyl) Transferase 3, Mucin Type	6.809
**GABRA2**	Gamma-aminobutyric Acid (Gaba) a Receptor, Alpha 2	6.791
**NCAM2**	Neural Cell Adhesion Molecule 2	6.704
**ANO3**	Anoctamin 3	6.597
**ADAMTS5**	Adam Metallopeptidase with Thrombospondin Type 1 Motif, 5	6.263
**CD55**	Cd55 Molecule, Decay Accelerating Factor for Complement (Cromer Blood Group)	6.159

FC represents fold change at q ≤ 0.05 of a gene following *h*HSS1 modulation compared to cells stably transfected with vector control.

**Table 2:** **37 most down-regulated genes following** ***h*** **HSS1 overexpression in U87 cells**

Symbol	Gene name	FC
**DHCR24**	24-dehydrocholesterol Reductase	-6.046
**FOS**	Fbj Murine Osteosarcoma Viral Oncogene Homolog	-6.103
**COL1A1**	Collagen, Type I, Alpha 1	-6.132
**PDK3**	Pyruvate Dehydrogenase Kinase, Isozyme 3	-6.236
**PGF**	Placental Growth Factor	-6.268
**CASC5**	Cancer Susceptibility Candidate 5	-6.276
**KIF11**	Kinesin Family Member 11	-6.342
**ERCC6L**	Excision Repair Cross-complementing Rodent Repair Deficiency, Complementation Group 6-like	-6.36
**KIF15**	Kinesin Family Member 15	-6.494
**SPC25**	Spc25, Ndc80 Kinetochore Complex Component, Homolog (S. Cerevisiae)	-6.902
**C7orf68**	Chromosome 7 Open Reading Frame 68	-7.093
**IGFBP1**	Insulin-like Growth Factor Binding Protein 1	-7.129
**FAM70A**	Family with Sequence Similarity 70, Member A	-7.265
**ESCO2**	Establishment of Cohesion 1 Homolog 2 (S. Cerevisiae)	-7.283
**PTPRF**	Protein Tyrosine Phosphatase, Receptor Type, F	-7.283
**GPR155**	G Protein-coupled Receptor 155	-7.323
**HIST1H2BM**	Histone Cluster 1, H2bm	-7.326
**NID1**	Nidogen 1	-7.326
**MKI67**	Antigen Identified by Monoclonal Antibody Ki-67	-7.88
**ELMO1**	Engulfment and Cell Motility 1	-7.918
**DOK5**	Docking Protein 5	-7.943
**FAM111B**	Family with Sequence Similarity 111, Member B	-7.975
**RRM2**	Ribonucleotide Reductase M2	-8.078
**MYBL2**	V-myb Myeloblastosis Viral Oncogene Homolog (Avian)-like 2	-8.361
**IGFBP3**	Insulin-like Growth Factor Binding Protein 3	-8.394
**SLFN11**	Schlafen Family Member 11	-8.461
**C4orf49**	Chromosome 4 Open Reading Frame 49	-8.636
**FAM115C**	Family with Sequence Similarity 115, Member C	-10.234
**ACPP**	Acid Phosphatase, Prostate	-10.234
**APLN**	Apelin	-10.699
**GLB1L2**	Galactosidase, Beta 1-like 2	-10.894
**TIMP3**	Timp Metallopeptidase Inhibitor 3	-10.898
**MT1M**	Metallothionein 1 m	-11.858
**BEND5**	Ben Domain Containing 5	-12.104
**TXNIP**	Thioredoxin Interacting Protein	-12.625
**HIST1H1A**	Histone Cluster 1, H1a	-15.458
**THBS1**	Thrombospondin 1	-18.526

FC represents fold change at q ≤ 0.05 of a gene following *h*HSS1 modulation compared to cells stably transfected with vector control.

The most up-regulated genes in U87 cells were interleukins and receptors (*IL1A, IL13RA2, IL1RN*), *CT45A5* from the cancer/testis (CT) family of antigens, and the cytoplasmic transporter *ATP6V0D2* (Table 1). The most down-regulated genes were thrombospondin 1 (*THBS1*) and histone cluster 1 (*HIST1H1A*). Among the most down-regulated genes in U87 is apelin (*APLN*), a ligand for the angiotensin-like 1 (APJ) receptor [7, 8] and a novel factor involved in angiogenesis (Table 2).

We identified 84 differentially expressed genes in A172 cells due to *h*HSS1 overexpression, when a lower FC cutoff of 1.5 was used (Table 3 and Table 4). Thus, overexpression of *h*HSS1 had a larger effect in U87 compared to A172 cells. *KRT15* and *MCM10* were the molecules with highest connectivity. Among the most up-regulated genes in A172 cells were zinc finger protein 22 (*ZNF2*2), keratin 81 (*KRT81*), the enzyme arylacetamide deacetylase (*AADAC*) and the extracellular protein amelotin (*AMTN*) (Table 3). The most down-regulated were the coiled-coil domain containing 102b (*CCDC102B*) and the pote ankyrin domain family member B (*POTEB*) (Table 4).

**Table 3:** **Total list of most up-regulated genes following** ***h*** **HSS1 overexpression in A172 cells**

Symbol	Gene name	FC
**C19orf63**	Chromosome 19 Open Reading Frame 63	11.881
**ZNF22**	Zinc Finger Protein 22 (Kox 15)	4.012
**KRT81**	Keratin 81	3.93
**AADAC**	Arylacetamide Deacetylase (Esterase)	3.317
**AMTN**	Amelotin	3.018
**JAM2**	Junctional Adhesion Molecule 2	2.66
**FAM133A**	Family with Sequence Similarity 133, Member A	2.606
**EDIL3**	Egf-like Repeats and Discoidin I-like Domains 3	2.524
**C2orf15**	Chromosome 2 Open Reading Frame 15	2.299
**CLDN1**	Claudin 1	2.239
**BICC1**	Bicaudal C Homolog 1 (Drosophila)	2.092
**IL2RG**	Interleukin 2 Receptor, Gamma	1.895
**SYTL5**	Synaptotagmin-like 5	1.887
**KAL1**	Kallmann Syndrome 1 Sequence	1.875
**CDH10**	Cadherin 10, Type 2 (T2-cadherin)	1.861
**SLC25A27**	Solute Carrier Family 25, Member 27	1.839
**TAF4B**	Taf4b Rna Polymerase Ii, Tata Box Binding Protein (Tbp)-associated Factor, 105 kda	1.837
**ACTA2**	Actin, Alpha 2, Smooth Muscle, Aorta	1.821
**NAP1L3**	Nucleosome Assembly Protein 1-like 3	1.795
**PLEKHA1**	Pleckstrin Homology Domain Containing, Family a (Phosphoinositide Binding Specific) Member 1	1.757
**IL18**	Interleukin 18 (Interferon-gamma-inducing Factor)	1.708
**KCTD16**	Potassium Channel Tetramerisation Domain Containing 16	1.689
**ZNF571**	Zinc Finger Protein 571	1.653
**INPP5A**	Inositol Polyphosphate-5-phosphatase, 40kda	1.643
**ZMAT1**	Zinc Finger, Matrin-type 1	1.642
**DOCK1**	Dedicator of Cytokinesis 1	1.617
**TSGA10**	Testis Specific, 10	1.598
**CADM1**	Cell Adhesion Molecule 1	1.592
**ECHS1**	Enoyl Coa Hydratase, Short Chain, 1, Mitochondrial	1.584
**ENTPD1**	Ectonucleoside Triphosphate Diphosphohydrolase 1	1.573
**ZRANB1**	Zinc Finger, Ran-binding Domain Containing 1	1.567
**PTPRE**	Protein Tyrosine Phosphatase, Receptor Type, E	1.548
**TP53INP1**	Tumor Protein P53 Inducible Nuclear Protein 1	1.543
**DUSP10**	Dual Specificity Phosphatase 10	1.543
**TM2D1**	Tm2 Domain Containing 1	1.527
**ZMAT3**	Zinc Finger, Matrin-type 3	1.522
**LTBP2**	Latent Transforming Growth Factor Beta Binding Protein 2	1.516

FC represents fold change at q ≤ 0.05 of a gene following *h*HSS1 modulation compared to cells stably transfected with vector control.

**Table 4:** **Total list of most down-regulated genes following** ***h*** **HSS1 overexpression in A172 cells**

Symbol	Gene name	FC
**MCM6**	Minichromosome Maintenance Complex Component 6	-1.501
**C6orf52**	Chromosome 6 Open Reading Frame 52	-1.501
**FERMT3**	Fermitin Family Member 3	-1.533
**SMC2**	Structural Maintenance of Chromosomes 2	-1.546
**SRPX**	Sushi-repeat Containing Protein, X-linked	-1.549
**SHCBP1**	Shc Sh2-domain Binding Protein 1	-1.564
**GPSM2**	G-protein Signaling Modulator 2	-1.564
**NES**	Nestin	-1.565
**SYCP2**	Synaptonemal Complex Protein 2	-1.575
**MCM10**	Minichromosome Maintenance Complex Component 10	-1.576
**EZH2**	Enhancer of Zeste Homolog 2 (Drosophila)	-1.58
**TMTC2**	Transmembrane and Tetratricopeptide Repeat Containing 2	-1.594
**FAM129A**	Family with Sequence Similarity 129, Member A	-1.596
**TMEFF2**	Transmembrane Protein with Egf-like and Two Follistatin-like Domains 2	-1.604
**CTSL2**	Cathepsin L2	-1.613
**ETV1**	Ets Variant 1	-1.614
**SGOL2**	Shugoshin-like 2 (S. Pombe)	-1.62
**ERCC6L**	Excision Repair Cross-complementing Rodent Repair Deficiency, Complementation Group 6-like	-1.621
**KRT15**	Keratin 15	-1.641
**SDPR**	Serum Deprivation Response	-1.656
**ACAT2**	Acetyl-coa Acetyltransferase 2	-1.7
**BDKRB1**	Bradykinin Receptor B1	-1.709
**CFI**	Complement Factor I	-1.711
**GPD2**	Glycerol-3-phosphate Dehydrogenase 2 (Mitochondrial)	-1.722
**TMOD1**	Tropomodulin 1	-1.729
**FAM64A**	Family with Sequence Similarity 64, Member A	-1.755
**ANO5**	Anoctamin 5	-1.782
**LRRC15**	Leucine Rich Repeat Containing 15	-1.812
**PAGE1**	P Antigen Family, Member 1 (Prostate Associated)	-1.822
**XRCC2**	X-ray Repair Complementing Defective Repair in Chinese Hamster Cells 2	-1.863
**EMP2**	Epithelial Membrane Protein 2	-1.868
**CD180**	Cd180 Molecule	-1.926
**ELOVL6**	Elovl Fatty Acid Elongase 6	-1.931
**PLCXD3**	Phosphatidylinositol-specific Phospholipase C, X Domain Containing 3	-1.938
**C7orf69**	Chromosome 7 Open Reading Frame 69	-1.941
**DMD**	Dystrophin	-1.947
**MNS1**	Meiosis-specific Nuclear Structural 1	-1.949
**FAM115C**	Family with Sequence Similarity 115, Member C	-2.005
**TEK**	Tek Tyrosine Kinase, Endothelial	-2.099
**CHRM3**	Cholinergic Receptor, Muscarinic 3	-2.122
**RGS16**	Regulator of G-protein Signaling 16	-2.144
**SULT1B1**	Sulfotransferase Family, Cytosolic, 1b, Member 1	-2.478
**ANKRD30B**	Ankyrin Repeat Domain 30b	-2.592
**B3GALT1**	Udp-gal:betaglcnac Beta 1,3-galactosyltransferase, Polypeptide 1	-2.841
**XIRP2**	Xin Actin-binding Repeat Containing 2	-3.387
**POTEB**	Pote Ankyrin Domain Family, Member B (includes others)	-6.162
**CCDC102B**	Coiled-coil Domain Containing 102b	-11.348

FC represents fold change at q ≤ 0.05 of a gene following *h*HSS1 modulation compared to cells stably transfected with vector control.

Fifteen genes were concordantly altered in both U87 and A172 cell lines, 14 were down-regulated (*JAM2, FAM115C, MNS1, ERCC6L, EMP2, EZH2, TMOD1, GPSM2, XRCC2, SGOL2, SMC2, FAM64A, MCM10, SHCBP1*), and 1 was up-regulated (*TAF4B*). Two genes were altered in different direction with *h*HSS1 overexpression: the complement factor I (*CFI*) was up-regulated in U87 cells (FC: 2.9) while it was down-regulated in A172 cells (FC:-1.7). Likewise, tek tyrosine kinase (*TEK*) was up-regulated in U87 (FC: 2.2) but it was down-regulated (FC:-2.1) in A172 cells.

### Network, pathway and functional analysis of genes influenced by *h*HSS1 overexpression in human U87 and A172 glioma cell lines

We evaluated the interaction and functional importance of the signaling pathways involving genes significantly modulated by *h*HSS1. The list of differentially expressed genes analyzed by IPA revealed significant networks and interactions. Figure 1 shows the top networks identified by IPA in both U87 and A172 cells. The highest significant network with 27 focus molecules and a significance score of 43 in the U87 cell dataset revealed genes related to the cell cycle, cell death, DNA replication, recombination and repair (Figure 1A). There was a significant up-regulation of *ANKRD1*, a nuclear factor that has negative transcriptional activity in endothelial cells [9]. Figures 1B shows the top network found in A172-*h*HSS1 clone #7. With a score of 48, the top network included molecules involved in cell cycle, cellular assembly and organization, DNA replication, recombination and repair. The highest significant network in A172-*h*HSS1 C#8 with a significance score of 50 revealed genes related to tissue morphology and cellular development (Figure 1C).

**Figure 1:** **Top molecular networks of genes up- and down-regulated in U87 and A172 cells overexpressing** ***h*** **HSS1.** Network of genes based on connectivity identified by IPA analysis. **A)** Top gene network of U87 cells depicting genes involved in cell cycle, cell death, DNA replication, recombination and repair. *ANKRD1* was the most up-regulated gene. Many genes with a direct and indirect relationship with *E2F* gene were down-regulated by HSS1. **B)** Top gene network of A172-*h*HSS1 C#7 showing genes involved in cell cycle, cellular assembly and organization, DNA replication, recombination and repair. Several genes down-regulated by *h*HSS1 in A172 C#7 cells are target genes regulated by *VEGF*. **C)** Top gene network of A172-*h*HSS1 C#8 showing genes involved in tissue morphology and cellular development. Some of the *h*HSS1 modulated genes in A172 C#8 cells are responsible for *ERK* regulation. Different shapes of the nodes (genes/gene products) represent the functional classes of the gene products and the lines represent the biological relationships between the nodes. The length of an edge reflects the evidence in the literature supporting that node-to-node relationship. The intensity of the node color indicates the degree of up- (red) or down-regulation (green) of the respective gene. Gray represents a gene related to the others that did not meet the cutoff criteria. A solid line without arrow indicates protein-protein interaction. Arrows indicate the direction of action (either with or without binding) of one gene to another.

The pathway analysis of U87 cells strongly suggest that *h*HSS1 modulates genes related to the role of *BRCA1* in DNA damage response (17 DEGs, *P* = 1.70e^−9^), ATM signaling (13 DEGs, *P* = 1.69e^−6^) and the mitotic roles of polo-like kinases pathway (14 DEGs, *P* = 2.53e^−6^). The top most significant pathway showed that 17 differentially expressed genes in U87 cells were related to the DNA damage response involving members of the BRCA family (Figure 2). *h*HSS1 down-regulated complexes of protein, namely BRCA1, BRCA2, Rad51, BARD and FANCD2 in U87 cells. These proteins are responsible for regulating the S and G2 phases of cell cycling. Genes involved in homologous recombination and chromatin remodeling were also down-regulated. The transcriptional regulator *E2F5* responsible for the G1/S phase transition was the only gene up-regulated in this pathway. The top 3 pathway in U87 cells regulated by *h*HSS1 was related to genes involved in the mitotic roles of polo-like kinases (Figure 3), which included genes involved in centrosome separation and maturation (*EG5, CDC2* and cyclin B), mitotic entry (*CDC25, PLK, CDC2* and *cyclin B*) and metaphase and anaphase transition (*APC, CDC20, PRC1, cyclin B, SMC1* and *Esp1*). Moreover, the functional analysis of differentially expressed genes in U87 cells, robustly suggested that *h*HSS1 affects the cell division process of chromosomes (57 DEGs, *P* = 7.75e^−25^), segregation of chromosomes (34 DEGs, *P* = 4.49e^−23^), mitosis (73 DEGs, *P* = 2.33e^−19^), M phase (45 DEGs, *P* = 1.53e^−17^), cell cycle progression (120 DEGs, *P* = 2.86e^−16^), cell death of tumor cell lines (141 DEGs, *P* = 1.80e^−15^) and proliferation of cells (235 DEGs, *P* = 2.23e^−15^).

**Figure 2:** **Role of BRCA in DNA damage response pathway is regulated by** ***h*** **HSS1-overexpression in U87 cells.** Blue color indicates down-regulation of a gene, orange color indicates up-regulation of a gene. This analysis was done using Ingenuity iReport.

**Figure 3:** **Mitotic roles of polo-like kinase pathway is regulated by** ***h*** **HSS1-overexpression in U87 cells.** Blue color indicates down-regulation of a gene, orange color indicates up-regulation of a gene. This analysis was done using Ingenuity iReport.

In A172 cells, the most significant pathways affected by *h*HSS1 overexpression were related to metabolism. Among them were butanoate and propanoate metabolism and the pathways related to valine, leucine and isoleucine degradation. The top most significant pathway was the butanoate metabolic pathway (A172-*h*HSS1 C#7: 5 DEGs, *P* = 4.35e^−5^; A172-*h*HSS1 C#8: 4 DEGs, *P* = 1.41e^−4^). Four genes were differentially expressed: *AADAC* and *ECHS1* were up-regulated while *ACAT2* and *ELOVL6* were down-regulated. The most affected biological processes in A172 cells were cell-cell contact (A172-*h*HSS1 C#8: 5 DEGs, *P* = 1.10e^−4^), growth of melanoma cell lines (A172-*h*HSS1 C#8: 3 DEGs, *P* = 1.49e^−3^) and migration of embryonic cell lines (A172-*h*HSS1 C#8: 3 DEGs, *P* = 2.25e^−3^). The biological process analysis was not determined for A172-*h*HSS1 C# 7.

### Validation of microarray data at the RNA level

For validation of microarray data, a sub-set of differentially expressed genes were selected corresponding to the highest fold-change and particularly those which were involved with proliferation, adhesion, migration and invasion. We assessed changes in gene expression using qRT-PCR for five different genes for each cell line: *CCDC102B, XIRP2, ANKRD30B, EDIL3* and *JAM2* for A172 cells evaluation; and the genes *IL13RA2, ANKRD1, APLN, NCAM2* and *THBS1* for U87 cells. From the genes selected for validation, only *XIRP2* showed a discrepancy in gene expression between qRT-PCR and microarray analysis for both A172 C#7 and C#8 clones (Figure 4).

**Figure 4:** **Validation of selected genes differentially expressed by** ***h*** **HSS1 overexpression in U87 and A172 cells.** Blue color indicates genes validated by qRT-PCR. Red color indicates genes differentially expressed by microarray analysis. **A)** Genes differentially expressed in U87 cells. **B)** Genes differentially expressed in A172-*h*HSS1 C#7 and **C)** A172-*h*HSS1 C#8.

### Effect of *h*HSS1 overexpression on cell cycle phases in human U87 and A172 glioma cell lines

We next evaluated the cell cycle phases in U87 and A172 cells in order to corroborate the microarray findings of differentially expressed genes in pathways related to cell cycle regulation. Previously we had shown that cell proliferation significantly decreased in cells overexpressing *h*HSS1 and observed a 5 and 10 hours delay in doubling time for U87 and A172, respectively [4]. The cell cycle analysis of day 4 and 5 from U87 and A172 cells respectively, showed a significant decrease of cells in phases G0/G1, while a significant increase in cells was seen in S and G2/M phases in U87 cells overexpressing *h*HSS1 (Figure 5). No difference in cell cycle distribution was observed for A172 cells, except for a significant decrease in S phase for A172-*h*HSS1 expressing cells compared with A172-wild type. Taken together, these results indicate that *h*HSS1 overexpression in A172 cells does not regulate a specific cell cycle phase but could prevent the overall progression of the cell cycle once it lead to a 10 hours delay in doubling time. This finding is consistent with the observed modulation of genes related to metabolic pathways.

**Figure 5:** **Effect of** ***h*** **HSS1 on cell cycle phases for glioma cells.** Cell cycle analysis in **A)** U87 cells and **B)** A172 cells. Cell cycle analysis was performed by propidium iodide staining followed by flow cytometry using day 4 and 5 from a U87 and A172 cell growth curve, respectively. Columns represent the mean percentage of cells in each phase of the cell cycle ± SEM (n = 2), *P* < 0.05, one way ANOVA with post hoc pairwise Tukey test.

### *h*HSS1 overexpression inhibits migration and invasion of human U87 and A172 glioma cell lines

One of the hallmarks of glioblastoma cells is that they infiltrate surrounding normal brain tissue and so lose constraints on cell migration. Our microarray analysis indicated that *h*HSS1 up or down regulated genes involved in cell migration, invasion and angiogenesis. To clarify an effect of *h*HSS1 on these key events involved in tumorigenesis, we used the modified Boyden chamber assay to study the migratory and invasive properties of U87 and A172 cells overexpressing *h*HSS1 (Figure 6). U87 cells overexpressing *h*HSS1 significantly lost their ability to migrate and invade through a matrigel matrix, compared to the U87-pcDNA.3.1 control cells. For A172 cells, C#7 but not C#8, showed a significant decrease in cell migration compared with the control. Moreover, *h*HSS1 had no effect on A172 invasion, indicating that overexpression of *h*HSS1 does not have a consistent effect on the migratory and invasive properties of A172 cells. Taken together, our data demonstrate that overexpression of *h*HSS1 decreases the invasive properties of U87 cells but has no effect on A172 cells.

**Figure 6:** **Overexpression of** ***h*** **HSS1 significantly affects the migration and invasion of glioma cells. A)** Transwell migration assay for U87 and A172 cells overexpressing *h*HSS1 or control vector. **B)** Matrigel invasion assay for U87 and A172 cells overexpressing *h*HSS1 or control. 10% FBS serum was added as chemoattractant. After 24 h incubation, cells that migrated through the membrane or invaded through the matrix were fixed, stained with H&E and pictures (200x, magnification) of 9 fields of each replicate was taken for cells counting. Two independent experiments using duplicates were done for each assay. Data shown are mean ± SEM. **P < 0.01; ***P < 0.001, *t*-test.

### *h*HSS1 overexpression by human U87 and A172 glioma cell lines inhibited tumor-induced migration and invasion of HUVEC

The migration and invasion of endothelial cells through basement membranes are crucial steps in the development of new blood vessels. Stimulation of endothelial cells by tumor cells is known for establishing an endothelial phenotype consistent with the initial stages of angiogenesis [10]. In order to determine if *h*HSS1 had an effect on angiogenesis, as suggested by our microarray analysis, we evaluated the ability of *h*HSS1 to impact these critical events in a co-culture assay. Glioma cells overexpressing *h*HSS1 and HUVEC were co-cultured in transwell chambers, and the tumor-induced migration and invasion of HUVEC through matrigel was estimated (Figure 7). At a 1:10 HUVEC:U87 ratio, there was a significant decrease in the invasion of HUVEC co-cultured with U87-*h*HSS1 cells compared to HUVEC co-cultured with U87-pcDNA3.1 control. However, overexpression of *h*HSS1 did not affect the migration of HUVEC cells co-cultured with U87 cells. It was previously reported that U87 cells promote morphogenetic changes in HUVEC, including the formation of net-like structures resembling neo-vasculature [10]. We noted that endothelial cells that invaded the matrix, in co-culture with U87-pcDNA3.1 control cells, appeared elongated with a narrower extended shape and aligned themselves to form net-like structures (Figure 7A, black arrow). In contrast, HUVEC co-cultured with U87-*h*HSS1 had a rounded or ‘teardrop-like’ morphology, and did not align themselves to form net-like structures (Figure 7A). HUVEC growing in co-culture with A172 C#7 and C#8 overexpressing *h*HSS1, displayed significant decrease in both migration and invasion ability when compared to HUVEC co-cultured with A172-pCDNA3.1 control cells (Figure 7B). These findings indicate that *h*HSS1 can impact angiogenesis, as it suppresses the tumor-induced HUVEC phenotype related to cell migration and invasion.

**Figure 7:** **Overexpression of** ***h*** **HSS1 impacts U87 and A172 tumor-induced HUVEC migration and invasion. A)** Transwell migration and invasion assay for HUVEC co-cultured with U87 cells overexpressing *h*HSS1 or control vector. **B)** Transwell migration and invasion assay for HUVEC co-cultured with A172 cells overexpressing *h*HSS1 or control vector. Glioma cells were seeded in the bottom chamber containing media with 2% FBS. After 24 h, media was changed to serum-free media supplemented with 0.1% BSA. HUVEC were seeded in the upper chamber containing media with 0.1% BSA. A172 or U87 cells were seeded at 10:1 ratio of HUVEC. After 24 h, cells that migrated and invaded the matrix were fixed, stained with H&E and pictures (200x, magnification) of 21 fields of each replicate were taken for cells counting. Two independent experiments using duplicates were done for each assay. Data shown are mean ± SEM. ***P < 0.001, *t*-test. Black arrow shows net-like formation of invaded cells.

### Purified *h*HSS1 protein inhibits *in vitro*angiogenesis

The migration and invasion of endothelial cells are essential for the formation of new blood vessels during neo-angiogenesis, and consequently are critical events for tumor growth. Because ectopic overexpression of *h*HSS1 in glioma-derived cells strongly inhibited HUVEC cell migration and invasion, we examined the effect of purified *h*HSS1 on the potential of HUVEC to form capillary-like structures. As shown in Figure 8, HUVEC growing on matrigel treated with vehicle control formed complex network of tubes after 8 h, which was inhibited and disrupted in a concentration-dependent manner by treatment with 500 nM or 200 nM of purified *h*HSS1.

**Figure 8:** **Purified** ***h*** **HSS1 inhibits HUVEC tube formation in a concentration-related manner.** HUVEC growing on top of matrigel were treated with different concentrations of purified *h*HSS1 or vehicle control (PBS). Cells were pre-treated with *h*HSS1-His protein or vehicle control for 3 h before plating on top of matrigel. After 8 h, cells were stained with crystal violet and tube formation was evaluated. Images (100x, magnification) are representative of two independent experiments done in duplicate. **A** and **C**) Inhibitory effect of purified *h*HSS1-His on tube formation using 500 nM and 200 nM of *h*HSS1 protein, respectively. **B** and **D**) Vehicle control was diluted following the protein dilution scheme.

### *h*HSS1 expression in GBM samples from the TCGA database

*h*HSS1 mRNA expression in 428 GBM samples from the TCGA database was compared to a list of 12 genes selected based on their involvement in GBM, invasion, migration, angiogenesis and significant pathways or networks identified from the U87/A172 cells overexpressing *h*HSS1. This analysis revealed a highly significant but weak inverse correlation with *BRCA2* (r = −0.224, *P* < 0.0005) (Figure 9A). Moreover, statistically significant inverse correlation with *ADAMTS1* (r = −0.132, *P* < 0.01) and direct correlation with endostatin (r = 0.141, *P* < 0.005) were found (data not shown). The subdivision of the GBM cohort based on high and low *h*HSS1 expression showed that the levels of *BRCA2* and *ADAMTS1* expression on *h*HSS1-high expression group are significantly lower compared to *h*HSS1-low expression group (*P* < 0.00006 and *P* < 0.014, respectively) (Figure 9B). Additionally, higher expression of endostatin was significantly found in *h*HSS1-high expression group compared to HSS1-low expression group (*P* < 0.048).

**Figure 9:** ***h*** **HSS1 expression analysis in GBM from the TCGA dataset. A)** Correlation analysis between *h*HSS1 and *BRCA2* expression (r = −0.224, *P* < 0.0005). **B**) Log2-transformed gene expression levels for selected genes between high and low-*h*HSS1 expression cohorts. Mean gene expression levels between cohorts were compared by two-tailed Student's t-test, *P* < 0.01. *P* values - HSS1 ^lo^ vs. HSS1 ^hi^ : (*h*HSS1, *P* < 6.55e^−98^), (*ADAMTS1*, *P* < 0.014), (*BRCA2*, *P* < 0.00006), Endostatin (*COL18A1), P* < 0.048).

## Discussion

In this study we have combined advanced bioinformatics with functional assays and subsequently identified key biological pathways directly or indirectly affected by *h*HSS1. The observed effect of *h*HSS1 included DEGs having either stimulatory or inhibitory effects, but ultimately leading to inhibition of tumoral and angiogenic properties. *h*HSS1 overexpression strongly affected a number of transcriptional regulators, enzymes, growth factors, transporters and extracellular matrix proteins, hence altering important signaling pathways, and impacting biological functions. The pathway analysis approach using IPA and Ingenuity® iReport indicated that *h*HSS1 plays a role in several biological functions considered hallmarks of cancer, including cell proliferation, cell cycle regulation, DNA replication, DNA repair, angiogenesis, cell migration, and cell invasion.

Previously, we have shown that *h*HSS1 overexpression negatively regulated proliferation of U87 and A172 cells [4]. Our microarray data of the same set of cells evaluated by pathway analysis yielded a similar effect of down regulation of genes involved in proliferation, cell cycle progression and cell division process. Furthermore, the cell cycle analysis demonstrated that the inhibition of U87 cell proliferation was accompanied by a decrease of cells in G0/G1 and a concomitant increase of cells in S and G2/M. The down regulation indicated by microarray analysis of *cyclin E, cyclin B, CDC2* and a complex of proteins (BRCA1, BRCA2, Rad51, BARD and FANCD2) responsible for regulating the S and G2 cell cycle phases, might partly explain the inhibitory effect of *h*HSS1 overexpression on proliferation previously reported for U87 cells.

The IPA top molecular network included *ANKRD1* as the most up-regulated gene in U87 cells, a nuclear factor that has negative transcriptional activity in endothelial cells [9]. There are indications that ANKRD1 (CARP) is a direct target of TGF-b/Smad signaling and acts as a negative regulator for cell cycle progression [11]. Thus, *h*HSS1 presumably could be targeting the TGF-b/Smad pathway via ANKRD1 up-regulation. Many genes with direct and indirect relationship with *E2F* gene were down-regulated by *h*HSS1. The *E2F* transcription factor family is known to play a central role in the expression of genes required for cell cycle progression and proliferation, particularly genes involved in DNA synthesis [12]. Thus, we can speculate that *E2F* play an important role in coordinating events associated with cell cycle arrest mediated by *h*HSS1. In parallel, *h*HSS1 regulated genes involved in centrosome separation and maturation (*EG5, CDC2, cyclin B*), mitotic entry (*CDC25, CDC2, Cyclin B, PLK*), metaphase and anaphase transition (*CDC, APC, PRC1, Cyclin B, Esp1, SMC1*), which could also have an effect on cell cycle and consequently cell proliferation. Conversely, *h*HSS1 overexpression in A172 cells does not seem to regulate a specific cell cycle phase. However, IPA and Ingenuity® iReport pathway analysis of A172 cells indicated that *h*HSS1 modulated genes related to metabolic pathways, which could in part have an effect over the global protein expression, thereby contributing to the regulation of proliferation. Thus, we can presume that *h*HSS1 mechanisms governing cell proliferation in A172 and U87 cells might be different. This difference may be explained based on the dissimilar deletions and genetic mutations linked to these cell lines [13].

It is worthy of note that *IL13RA2* was the most up-regulated gene induced by *h*HSS1 in U87 cells. The *IL13RA2* gene is often overexpressed in brain tumors [14] and is involved in the invasion and metastasis of ovarian cancer cells [15]. Overexpression of the IL13RA2 chain in human breast cancer cell line and pancreatic cancer cell line inhibited tumor development in nude mice, probably mediated by IL-13 [16]. *IL13RA2* overexpressing tumor cells produced high levels of IL-8 which has been shown to reduce tumorigenicity in several tumor models [16–18]. Decreasing the expression of the IL-13 receptor also leads to an increasing tumorigenicity [16].

Overexpression of *h*HSS1 affected the migratory and invasive properties of U87 cells induced by FBS as a chemoattractant. In A172 cells, IPA top molecular network analysis showed that several genes down-regulated by *h*HSS1 are target genes regulated by VEGF or genes responsible for ERK regulation. However, we did not observe *in vitro* a consistent negative regulation of A172 stable clones migratory or invasive proprieties induced by *h*HSS1. Variations in migratory and invasive proprieties induced by *h*HSS1 in different glioma cell lines are likely due to diverse genetic background (e.g. mutations and deletions) [13], probably involving other signaling pathways and molecules.

Our data however, showed that A172 glioma-derived cells overexpressing *h*HSS1 significantly inhibited HUVEC migration and invasion in low-serum protein conditions, indicating an indirect functional role for *h*HSS1 in angiogenesis. Moreover, in the same cell culture conditions, U87 cells overexpressing *h*HSS1 inhibited invasion but not migration of HUVEC cells. It has been previously reported that stimulation of endothelial cells by tumor cells establishes an endothelial phenotype consistent with the initial stages of angiogenesis [10, 19]. Although U87-overexpressing *h*HSS1 cells did not inhibit HUVEC migration, restraint of relevant morphological changes indicative of early angiogenesis were noted in HUVECs that invaded the matrix (i.e. HUVECs did not align themselves to form net-like structures relative to the control cells). Inhibition of net-like formation of HUVEC in co-cultures is consistent with the action of angiogenesis inhibitors like angiostatin and endostatin [10]. Additionally, we found that treatment of HUVEC cells with purified *h*HSS1, efficiently inhibited HUVEC tube formation ability, indicating that there is a direct functional relation between *h*HSS1 and HUVEC cells. Further mechanistic studies are required to determine how *h*HSS1 inhibits tube formation. However, our microarray data of U87 glioma cells indicated that *h*HSS1 down-regulated genes involved in angiogenesis, including *THBS1* and *APLN*. THBS1 is reported to stimulate or inhibit cell adhesion, proliferation, motility and survival in a context-dependent and cell-specific manner [20]. Although THBS1 is a potent inhibitor of angiogenesis, N-terminal proteolytic and recombinant peptides related to THBS1 have clear pro-angiogenic activities mediated by beta-1 integrins [21]. Moreover, glioma cell lines secrete significant levels of THBS-1, and high levels of THBS1 have been found in glioma tissues [22, 23]. Among the most down-regulated genes in U87 is *APLN*, a ligand for the angiotensin-like 1 (APJ) receptor [7, 8]. *APLN* expression has been observed to be highly up-regulated in the microvasculature in brain tumors. In particular, *APLN* has been shown to be needed for intersomitic vessel angiogenesis and the promotion of angiogenesis in brain tumors [24]. It is of further interest that *ADAMTS5* was among the highly up-regulated genes. ADAMTS5 is a metalloproteinase with the ability to slow tumor growth and diminish tumor angiogenesis, together with reduced tumor cell proliferation and increased tumor cell apoptosis [25]. The fact that *h*HSS1 strongly down-regulates *THBS-1* and *APLN*, and highly up-regulates *ADAMTS5* in the *h*HSS1-overexpressing cells is consistent with the observed *in vitro* results where angiogenesis was greatly suppressed by purified *h*HSS1. It is important to note that the GBM TCGA database analysis did not show a significant correlation between *hHSS1* and the expression of *APLN* and *THBS-1* genes, as observed for the microarray analysis using U87 *hHSS1*-overexpressing cells. This discrepancy could be due to potentially lower expression levels of *h*HSS1 in tumor tissues (not higher than 3.5-fold relative to normalization controls) compared to U87 cells ectopically overexpressing *h*HSS1 (11.7-fold). In addition, most of the 12 genes evaluated were expressed in the tumor tissue at relatively lower levels than 3.5-fold.

It was recently suggested that *BRCA1-2* carriers present higher expression of angiogenic factors VEGF, HIF-1a and higher microvessel density than in sporadic cancers [26], thus providing a link between *BRCA* genes and angiogenesis. Interestingly, the analysis of GBM dataset from TCGA revealed a highly significant inverse correlation between *h*HSS1 and *BRCA2* expression, and that the levels of *BRCA2* expression on HSS1-high gliomas were also significantly lower than on HSS1-low expression gliomas. This finding is intriguing in light of tube formation data that suggested purified *h*HSS1 inhibits HUVEC tube formation, thus implicating a role of *h*HSS1 in angiogenesis. It has been shown that *BRCA2*-defective cancer cells or treatment of cancer cells with *BRCA2* siRNA significantly reduces *BRCA2* protein and mRNA expression, leading to tumor radio-sensitization *in vitro* and *in vivo*, mainly through the inhibition of homologous recombination repair [27, 28]. Moreover, knockdown of BRCA2 greatly sensitizes glioma cells to DNA double strand breaks and the induction of cell death following temozolomide and nimustine treament [29].

*ADAMTS1* is a protease commonly up-regulated in metastatic carcinoma. *ADAMTS1* processing of versican is important in cell migration during wound healing and endothelial cell invasion [30, 31]. In addition, up-regulation of *ADAMTS1* in tumors participate in the remodeling of the peritumoral stroma, tumor growth and metastasis [32]. Our analysis from the TCGA database suggest a significant inverse correlation between *h*HSS1 and *ADAMTS1* expression, which is consistent with a role of *h*HSS1 in inhibition of tumor growth, progression and metastasis. GBM from TCGA also revealed a significant positive correlation between *h*HSS1 and endostatin (*COL18A1*) expression. Endogenous expression of endostatin by C6 glioma cells result in a reduced tumor growth rate *in vivo* that is associated with inhibition of tumor angiogenesis [33]. Further studies are required to clarify a correlation between a down-regulatory effect of *h*HSS1 on *BRCA2* and *ADAMTS1* genes as well as a direct correlation between *h*HSS1 and endostatin. However, our data suggest that *h*HSS1 could also potentially be developed as an adjuvant therapy for the effective treatment of gliomas.

It was reported that endostatin blocks VEGF-induced tyrosine phosphorylation of KDR/Flk-1 and activation of ERK, p38 MAPK, and p125FAK in human umbilical vein endothelial cells [34]. IPA top molecular network analysis in A172 cells showed that several genes down-regulated by *h*HSS1 are target genes regulated by VEGF or genes responsible for ERK regulation. Development of endostatin has been undertaken for the treatment of gliomas based on extensive preclinical data [35]. The mechanism of action focused on inhibition of angiogenesis highlights the possibility of combining *h*HSS1 and endostatin in the potential treatment of glioma. A potential synergistic effect could even lead to dose reductions in the level of administered therapeutic agent.

Angiogenesis is a complex process that involves the activation, proliferation, migration and invasion of endothelial cells to form new capillaries from existing blood vessels. The endothelial cells involved in tumor development dissolve their surrounding extracellular matrix, migrate toward the tumor, proliferate and form a new vascular network [36]. The anti-angiogenic effect of *h*HSS1 seems to correlate with the effect of the potent angiogenesis inhibitor endostatin [37], in that both proteins are extracellular proteins with the ability to negatively regulate HUVEC cell migration, invasion, tube formation as well as invasion of tumor cells [38].

## Conclusions

It has been proposed that the ideal cancer-therapy should be directed at two distinct cell populations, a tumor cell population and an endothelial cell population, each of which can stimulate growth of the other [39, 40]. Combined treatment of each cell population may be better than treatment of either compartment alone [41]. Our microarray and *in vitro* data suggest that *h*HSS1 protein is involved in the negative regulation of fundamental biological processes such as cell proliferation, migration, invasion, tumorigenesis and angiogenesis. Therefore, *h*HSS1 could be a potential therapeutic to target not only glioma tumor cells growth, but also endothelial cell neo-vascularization, and could provide a novel therapeutic intervention along with chemotherapy.

## Abbreviations

DEGs: Differentially expressed genes
ER: Endoplasmic reticulum
FC: Fold-change
IPA: *h*HSS1: Human hematopoietic signal peptide-containing secreted 1
HUVEC: Human umbilical vein endothelial cells
IPA: Ingenuity pathway analysis
GBM: Glioblastoma
TCGA: The cancer genome atlas.
